The article "Comprehensive Medical Analysis of Clinical Diseases and Syndromes Based on Rheumatoid Factor Interfering Immune Blood Cell Damage" was retracted in 2023. Reason: concerns about the peer review.

# Comprehensive Medical Analysis of Clinical Diseases and Syndromes Based on Rheumatoid Factor Interfering Immune Blood Cell Damage

**DOI:** 10.1155/2021/2290650

**Published:** 2021-06-29

**Authors:** Hui Zhu

**Affiliations:** ^1^Department of Rheumatology and Immunology, The First Hospital of Qiqihar, Qiqihar, Heilongjiang 161000, China; ^2^Affiliated Qiqihar Hospital, Southern Medical University, Qiqihar, Heilongjiang 161000, China

## Abstract

Rheumatoid arthritis bothers people. According to statistics, the prevalence of rheumatoid arthritis represents about 3% of the world's population. Rheumatoid factors can interfere with immune blood cells, which is very harmful to human health. In order to solve the damage of rheumatoid factor to health and study its influence on immune blood cells, this paper constructs a case template through case investigation of rheumatoid arthritis patients and creates damage assessment matrix by using comprehensive quantitative and qualitative analysis. The horizontal coupling degree between rheumatoid factor and interference of blood cell system is investigated, and the relationship between them is studied. The experimental results show that there is a correlation between rheumatoid factor and immune blood cells, the correlation coefficient is 0.87, the presence of rheumatoid factor in blood cells, and the cell system damage rate is about 30% higher than that without rheumatoid factor; the study found that there is a great difference in the age of rheumatoid factor in the population, and the age of patients is generally above 45 years old. This shows that rheumatoid factor can cause great damage to immune blood cell system and affect people's health level.

## 1. Introduction

As an inflammatory agent caused by bacteria, viruses, and other pathogens, rheumatoid factor is the leading cause of rheumatoid arthritis. Chronic multiple arthritis is the main clinical manifestation of rheumatoid arthritis. Chronic synovial inflammation and pannus formation in the lesion can lead to the destruction of articular cartilage and bone, and finally, the joint deformity and function are lost. In addition, rheumatoid arthritis can also significantly increase or promote the mortality of cardiovascular and other diseases. Therefore, rheumatoid arthritis is a very serious harm to human health, with a high morbidity and mortality. It has been reported that the occurrence of rheumatoid arthritis is mostly related to air pollution, heredity, infection, and autoimmune factors, but the exact mechanism is still unclear [1]. There are many pathological factors in the local area of rheumatoid arthritis, among which clot formation is considered as one of the indicators for the diagnosis of rheumatoid arthritis. Angiogenesis is the material structure basis of pannus formation, which can enrich a variety of inflammatory cells, promote the proliferation of synovial cells, make articular cartilage and bone suffer erosion and damage, and then mediate the occurrence and development of rheumatoid arthritis [2].

Rheumatoid arthritis is a common autoimmune disease in rheumatism. Its main manifestation is chronic multijoint synovitis, then pannus formation, and finally joint and bone destruction. The main pathological manifestations of rheumatoid arthritis are lymphocyte infiltration and synovial cell proliferation. With the progress of the disease, pannus appears, destroying the normal structure of cartilage and bone and eventually leading to joint deformity and dysfunction [3]. The incidence rate of rheumatoid arthritis is about 2.7% in China and 3% in the world. The incidence of female patients is higher than that of men. It can occur at all ages, but the peak age is 30–50 years old. Rheumatoid arthritis can not only lead to systemic joint dysfunction, but also often involve other systems including heart, lung, kidney, blood system, and so on [4]. Among them, the damage of immune blood cell system is very serious, which will eventually lead to inflammation and pathological process, including promoting synovial inflammation, pannus formation, joint erosion, and destruction. Based on the protection of human rights to life and health, experts at home and abroad have conducted numerous studies on the damage of rheumatoid factor to the immune system of blood cells [5].

Ren et al. studied the role of autoimmunity in the early stage of resistance to rheumatoid arthritis from the perspective of human autoimmunity. Through clinical research on patients, he compared serum antibody, positive, specificity, and sensitivity between patients with rheumatoid arthritis and normal people. Through data, it was proved that human immunity has important significance for the prevention and treatment of rheumatoid arthritis [6].

Liao et al. through the establishment of a control experimental group, the patients with rheumatoid arthritis research, and statistical data in the study found that patients with rheumatoid arthritis after treatment; its rheumatic factor, reactive protein and immunoglobulin have a significant decline, it concluded that rheumatoid arthritis and human rheumatic factor, reactive protein, and immunoglobulin have a certain relationship. The data of these three items can be used in the detection of rheumatoid arthritis [7].

Wang et al. think that rheumatoid factor will directly affect the immune blood cell system. Therefore, in order to evaluate the effect of rheumatoid factor, the serum samples containing rheumatoid factor with different dilution degree were determined by experiment. By establishing the calculation template, the influence of different content of rheumatoid factor on blood cell system was calculated, and the interference of rheumatoid factor on serum was determined [8].

The above research has a specific reference value for the intervention of rheumatoid factor in the immune cell system, but due to the small statistical data, statistical methods, and calculation methods, there are some differences between the results and the actual situation [9]. This paper analyzes the advantages and disadvantages of previous studies and then proposes a new model of immune cytokine network based on the above two models. This paper mainly describes the model from two aspects: the basic characteristics of the model and the composition of the model [10]. The composition of the model includes the grid, individual definition, state, action definition, and individual [11].

## 2. Methods of Interfering Immune Blood Cells with Two Kinds of Rheumatic Factors

### 2.1. Rheumatoid Factors

Rheumatoid factor (RF), as an inflammatory factor caused by bacteria, viruses, and other pathogens, is the main cause of rheumatoid arthritis. Chronic multiple arthritis is the main clinical manifestation of rheumatoid arthritis. Chronic synovial inflammation and pannus formation in the lesion can lead to the destruction of articular cartilage and bone, and finally, the joint deformity and function are lost. In addition, rheumatoid arthritis can also significantly improve or promote the mortality of cardiovascular and other diseases. Therefore, rheumatoid arthritis is a disease with high morbidity and mortality, which is extremely harmful to human health. It has been reported that the occurrence of rheumatoid arthritis is mostly related to air pollution, heredity, infection, and autoimmune factors, but the exact mechanism is still unclear. There are many pathological factors in the local area of rheumatoid arthritis, among which the formation of pannus is considered as one of the markers to determine rheumatoid arthritis. Angiogenesis is the material structure basis of pannus formation, which can enrich a variety of inflammatory cells, promote the proliferation of synovial cells, and make articular cartilage and bone suffer erosion and damage, and then mediate the occurrence and development of rheumatoid arthritis [12].

Clinical medical case information management system is a platform for information system to store and process unstructured data efficiently. It can use tree structure to organize all kinds of data required by website, including multimedia resources. The construction and implementation of a clinical case information management system will be able to solve the query, storage, and import of different unstructured data. It provides perfect data processing services for the application system connected to the system, so as to solve the problem that the unstructured data of enterprises cannot be efficiently processed [13].

Rheumatoid arthritis (RA) is an autoimmune disease characterized by synovitis. Its FLS has been proved to be the key to the development of inflammation and joint injury in rheumatoid arthritis. The main physiological function of normal FLS is to nourish and lubricate articular cavity and cartilage and also participate in cartilage metabolism. However, in rheumatoid arthritis, compared with normal synovial cells, FLS has abnormal morphology and a large number of hyperplasia abnormalities. Before the typical clinical manifestations of rheumatoid arthritis, FLS can be activated by the interaction between soluble factors and cell surface. These stimulating factors include some infectious or noninfectious antigens and their products. Thus, a large number of cytokines are released, which leads to joint inflammation and bone destruction [14]. The main pathological changes of rheumatoid arthritis focus on synovium and synovial associated cells. At present, researches on rheumatoid arthritis mainly focus on interleukin family, tumor necrosis factor family, and other related cytokines [15].

Synovitis and bone erosion are the two most important basic features in the pathological process of rheumatoid arthritis. FLS is the most important target cell among all the cells involved in the pathological changes and development of rheumatoid arthritis. In general, there are only 1-2 layers of cells in synovial joint, which can secrete synovial fluid for lubrication and protection. However, in patients with rheumatoid arthritis, the thickness of synovial lining layer at the boundary of joint cavity can be increased to 10–15 layers of cells, among which type A cells have macrophage-like function and type B cells have fibroblast-like function. In addition to morphological changes, the proliferation of rheumatoid arthritis FLS was enhanced. In the acute stage of rheumatoid arthritis, the subsynovial membrane is mainly exudative and infiltrative, leading to endothelial cell enlargement, interstitial edema, small vessel dilatation, and neutrophil infiltration. With the progress of the disease, the synovium gradually thickens and forms villous protuberances, which can adhere to the articular cartilage, invade the cell matrix, secrete a large number of matrix metalloproteinases, aggravate the destruction of cartilage and bone, and significantly enhance the ability to secrete inflammatory cytokines and adhesion molecules [16].

Rheumatoid arthritis, characterized by erosive arthritis, is a systemic autoimmune disease with a high prevalence rate. Its pathological damage can damage the cartilage and bone of the joint and eventually be reflected in the deformity of the joint and even the loss of function. In addition, rheumatoid arthritis can greatly increase the mortality of cardiovascular and other diseases. Rheumatoid arthritis (RA) is a kind of disease which is extremely harmful to human health and has a high disability and mortality rate [17]. There are many kinds of pathological factors in the local area of rheumatoid arthritis, among which inflammatory lesions and pannus formation are considered to be the most important ones. Angiogenesis is not only the material structure basis of pannus formation but also can enrich a variety of inflammatory cells, promote inflammatory lesions, and then mediate the occurrence and development of rheumatoid arthritis. Therefore, the study of angiogenesis inducing factors has become the focus of many scholars. As the most important angiogenic stimulant, vascular endothelial growth factor plays an essential role in the onset and development of rheumatoid arthritis [18].

### 2.2. Immune System

The immune system is not only the mechanism of the human body to complete the immune function, but also the organization for the immune response. It is also a natural protection barrier for the human body to resist the external pathogens [15]. It can prevent and eliminate the invasion of foreign bodies such as foreign viruses timely and effectively. It is a very complex system composed of immune tissues, immune organs, immune cells, and immune molecules. The research on immune system includes theoretical immunology and artificial immune system. Theoretical immunology (including computational immunology) is mainly used to explain all kinds of phenomena in immunology, and it can be used to solve the problems in immunology or medicine. One of the main research directions of theoretical immunology is computational immunology. Computational immunology generally uses nonlinear theory, differential equation, and computer simulation to model the human immune system. By analyzing the model, various phenomena and different mechanisms of human immune system are explained. Artificial immune system explores the nature and mechanism of human immune system in science and engineering, so as to find new ways to deal with science and engineering. However, theoretical immunology and artificial immune system do not develop independently, but promote each other and develop together. In fact, the modeling and simulation of human immune system is not only a part of theoretical immunology but also a part of artificial immune system [15].

Immune cytokine network has the characteristics of diversity and repeatability, so the research on this aspect of immune cytokine network is always very complex, so it is difficult for researchers to have a consistent specification in the description and modeling of immune cytokine network. At present, research on the cytokine immune network is not only a research point in the biological field, but also a research difficulty in the biological field. Although many people have done extensive research and research on the immunocytokine network and at the same time obtained many important research results, there are still many problems that have not been effectively resolved [19]. Researchers have done a lot of research on one kind of cytokines, involving only a single cytokine, and less on the integrity of the immune cytokine network. However, the cytokines secreted by immune cells are not unconnected. They are interconnected through the regulation of immune cells. Therefore, it is very important to study the integrity of immune cytokine network [20]. At present, the general model is

(1) $$\begin{array}{c} \sum_{n=1}^{i}\left(\vartheta r_{n}*w_{n}r_{n}+\vartheta \mu_{n}j_{n}\mu_{n}\right)-\sum_{j=1}^{i}\vartheta \theta_{n}\nu_{n}-\vartheta r_{i}*S_{i}=Q, \end{array}$$

among which,

(2) $$\begin{array}{c} \vartheta =\frac{6}{5\left(a_{i}+a_{j}\right)}{\left[\frac{r_{i}r_{j}}{r_{i}+r_{j}}\right]}^{1/2}. \end{array}$$

The parameters are AI and AJ

(3) $$\begin{array}{c} a_{n}=\frac{1-t_{n}^{2}}{S_{n}}\;\left(n=i,j\right). \end{array}$$

At present, the research on the immune system is not thorough enough. Researchers have only focused on individual cytokines and have not conducted a detailed and in-depth study on the integrity of cytokines. However, these cytokines are not unconnected. Therefore, researchers should pay more attention to the overall immune characteristics emerging from immune cytokine networks. Secondly, in previous research methods, most researchers use manual experiments. However, the biggest drawback of manual experiments is that it is difficult to study complex networks such as immune cytokine networks. Therefore, we cannot simply rely on manual experiments; finally, due to the limitations of modern science and technology on the immune cytokine network and the variety of cytokines themselves, so far there is no relatively perfect immune cytokine network model [21].

The role of immune blood cells as immune monitoring cells has been widely concerned in autoimmune diseases. Most scholars believe that immune blood cells play a protective role and prevent the onset of autoimmune diseases. It can help patients with hematological remission and reduce the recurrence rate, but at the same time, the incidence of infection and second tumor is also significantly increased [22]. This brings about not only great difficulties to the treatment but also huge economic burden to the families of patients. With the development of cell biotechnology, autologous cell transfusion is benefiting more patients with hematologic diseases. Therefore, more attention has been paid to the role of immune cells in the disease, because it is the cornerstone of cell biological therapy in the future.

### 2.3. Clinical Medical System

With the rapid development of digital medicine, electronic health data is growing rapidly. How to make full use of huge medical and health data to improve the level and quality of medical and health services is one of the hottest issues in current research [23]. In the hospital information system, the same medical term has many different forms of reference, which seriously hinders the integration and utilization of medical data. It is the premise of medical data integration and utilization to map various medical terms to standard medical terms, namely, medical terminology standardization or medical entity link. In the medical field, diversity is the most common phenomenon, and the research focus of entity standardization is focused on solving the problem of entity diversity. The existing entity standardization methods usually use entity context information for entity disambiguation and use the similarity between entity reference and entity concept to solve the problem of entity representation diversity [24].

At present, a large number of isolated disease entities are stored in the medical outpatient database of the medical system, without context information. The single medical entity has various forms and serious nonstandard problems. The common method to solve the problem is the edit distance algorithm. This paper attempts to construct the synonym knowledge base of medical disease entity, and then according to the diversity of single medical entity form, on the basis of existing methods, try to use the machine learning method with a small amount of manual intervention and high accuracy, and according to the information of patients, solve the problem of single medical entity link from three levels: record level, patient level, and hospital level. To this end, we set up a relevant calculation template [25].

The number of positive and negative examples of a template can be used to calculate the accuracy rate of creating the target entity to normalize the entity. The more positive examples, the more general the editing changes captured by the pattern, the better the pattern with more positive examples and few or no counterexamples. Let *X* be the number of positive examples and *I* the number of counterexamples. According to the *Y* estimation criterion, a score value is used to measure the mode. The larger the score, the better the editing mode [26].

(4) $$\begin{array}{c} M=\frac{x}{\left(x+i+1\right)}. \end{array}$$

According to the characteristics of the medical system, we improve the relevant calculation function:

(5) $$\begin{array}{c} f\left(i\right)=x_{0}+x_{1}y_{1}+x_{2}y_{2}+x_{3}y_{3}, \end{array}$$

where *x* is the cosine similarity, *y* is the adjacency degree, *I* is the page ranking value, and 0, 1, 2, and 3 are the weight parameters.

(6) $$\begin{array}{c} W=\frac{N_{1}r_{2}^{2}}{2}+\frac{N_{2}r_{2}^{2}}{2}+N_{2}d_{2}^{2}+\left(\frac{N_{3}r_{3}^{2}}{2}+N_{3}d_{3}^{2}\right)*0.1+\frac{2}{3}N. \end{array}$$

### 2.4. Coupling Relationship

Coupling theory is the main theory of this paper. The term “coupling degree” first appeared in physics. It originally refers to the measurement of the degree of correlation between circuit modules. Initially, it was used mainly in engineering research such as communication and machinery and then introduced in economic research. Coupling refers to the dynamic common relationship of mutual restriction or promotion or evolution formed by multiple narrow systems or modes of movement through various interactions and influences [27]. The coupling system composed of multiple subsystems has the characteristics of integrity, relevance, diversity, and coordination [28]. The integrity refers to the combination of different subsystems according to the new movement law; the correlation refers to the interaction between subsystems and the existence of different degrees of correlation; diversity refers to the influence of different subsystems according to different needs. Coordination means that the coupling subsystems are recombined with the changes of different factors, resulting in the diversity of coupling systems and the enhancement of coordinated development between systems [29]. In short, coupling degree describes the degree of interaction and interaction among different subsystems in the same coupling system [30].

Suppose the variable is the order parameter of rheumatoid factor immune blood cell system, which is the B index of the *a*-order parameter. Rheumatoid factor and immune blood cells are completely different but interact with each other. In general, the contribution of order parameters in subsystems to the degree of system ordering can be realized by integration methods such as linear weighting method.

(7) $$\begin{array}{c} m_{a}=\sum_{b=1}^{n}\lambda_{ab}\vartheta_{ab}. \end{array}$$

Among them, *a* is the contribution degree of subsystem to the ordering degree of rheumatoid factor immune blood cell system, and *b* is the weight of each sequence parameter.

Let *m*_1_ and *m*_2_ represent the changes of rheumatoid factor and immune blood cell system, respectively, and their changes are represented by *m*_1_ and *m*_2_, respectively. In this paper, the dispersion coefficient is used to represent the coordination degree between rheumatoid factor M1 and immune blood cell system *m*_2_, reflecting the variation or dispersion between them. The smaller the coefficient is, the greater the degree of coordination is. The formula for calculating the coefficient *Q* is as follows:

(8) $$\begin{array}{c} Q=2{\left(1-\frac{m_{1}m_{2}}{{\left[\left(m_{1}+m_{2}\right)/2\right]}^{2}}\right)}^{1/2}. \end{array}$$

The smaller the *Q* value, the higher the coordination between immune blood cells and rheumatoid factor. When *Q* = 0, the difference between the two systems is the smallest, and *m*_1_ and *m*_2_ coscheduling is the highest. Therefore, *Q* can be used as an index to measure the coupling degree of *m*_1_ and *m*_2_.

The coupling degree model is established as follows:

(9) $$\begin{array}{c} Q_{n}={\left\{\frac{\left(m_{1}*m_{2}\ldots m_{n}\right)}{\left[\pi \left(m_{s}+m_{k}\right)\right]}\right\}}^{1/n}. \end{array}$$

For the convenience of analysis, the coupling function *Q* of rheumatoid factor and immune blood cells can be expressed as follows:

(10) $$\begin{array}{c} Q=\frac{2{\left(m_{1}*m_{2}\right)}^{1/2}}{\left(m_{1}+m_{2}\right)}. \end{array}$$

## 3. Interference of Three Rheumatic Factors on Immune Blood Cell System

### 3.1. Research Object

The clinical data (gender, age of visiting or diagnosis, clinical symptoms, and signs at admission) were collected from 100 patients with blood immune system damage caused by rheumatoid factors in a city hospital. The auxiliary examinations included detection of respiratory virus antigen, detection of T lymphocyte subsets, detection of allergens, bronchoscopy, BALF cell count, and lung function. Follow-up was made by telephone and outpatient visits. The collected data were analyzed retrospectively and the conclusion was drawn, as shown in Figure 1.

### 3.2. Purpose of the Experiment

Through the follow-up investigation of patients, the influence of rheumatoid factor on immune blood cell system was understood. After treatment, if rheumatoid arthritis is effectively controlled and if the control effect is obvious were investigated [31]. The objective is to study the comprehensive medical system of clinical diseases and syndromes in which rheumatoid factor interferes with immune blood cell system damage, so as to provide reference for the treatment of immune blood cell system caused by rheumatoid factor.

### 3.3. Data Statistics

SPSS19.0 was used for all data analysis and double-sided test was used for statistical test. Significance was defined as 0.05, and *P* < 0.05 was considered as a statistically significant difference. The statistical results were shown as mean ± standard deviation (*x* ± SD). When the test data obeyed normal distribution, double-sided *t*-test was used within the group, and independent sample *t*-test was used between groups. If the routine distribution is insufficient, two separate samples and two related samples will be used for inspection. The calculation formula is as follows:

(11) $$\begin{array}{c} P=\sqrt{\frac{\sum_{a=1}^{a=x}{\left(Rf\left(W\left(\gamma_{a}\right)\right)-Rf\left(W_{0}\left(\gamma_{a}\right)\right)\right)}^{2}}{\sum_{a=1}^{a=x}{\left(RfW_{0}\left(\gamma_{a}\right)\right)}^{2}}}. \end{array}$$

## 4. Analysis of Four Rheumatic Factors Interfering Immune Blood Cell System

### 4.1. Distribution of Patients with Rheumatoid Factor

Based on the investigation of 100 patients, we have made statistics on the age and gender of patients. The specific distribution is shown in Table 1 and Figures 2 and 3.

From the chart, we can clearly see that the majority of patients with rheumatoid factor are over 45 years old, reaching 69%. Overall, male patients are much higher than female patients. Among 100 patients, 62 are men and 38 are women, 24% higher. It can be found that patients with rheumatoid factor over 45 years old are more likely to suffer from rheumatoid factor [32].

### 4.2. Changes of Immune Blood Cells before and after Treatment

We made statistics on the changes of immune blood cells before and after treatment to determine the damage degree of rheumatoid factors on immune blood cell system. We counted the contents of hemoglobin, red blood cells, and platelets in blood. The specific data are shown in Table 2 and Figures 4 and 5.

The graph shows that after treatment, hemoglobin, red blood cells, platelets, and rheumatoid factors in patients's immune cells have a significant reduction, among which the decrease in hemoglobin is the most obvious [33]. This shows that rheumatoid factor is the main factor affecting rheumatoid arthritis, and reducing rheumatoid shutdown factor can effectively treat rheumatoid arthritis.

### 4.3. Antibody Changes before and after Treatment

In order to understand whether the patients produce antibodies to rheumatoid factor after treatment, we also conducted corresponding research and statistical data, as shown in Table 3 and Figure 6.

It can be seen from the diagram that after treatment, the number of antibodies and the number of patients' antigens have changed to some extent, including the number of antibodies increasing by almost 40% and the number of antigens by about 20%. This shows that after treatment, the resistance of patients to rheumatoid factors has improved to a certain extent, but from the perspective of cure, the effect is not particularly ideal.

### 4.4. Degree of Blood Cell Damage

We have carried out the corresponding investigation on the patient's blood cell damage and the quantification processing through the related calculation way; we obtained the patient immune blood cell system damage *P* value, as shown in Table 4 and Figure 7.

It can be seen from the chart that rheumatoid factor has obvious damage effect on immune blood cell system, but after treatment, immune blood cells can basically recover to the original level, which means that the immune blood cell damage caused by rheumatoid factor can be recovered through treatment, which plays an important role in diseases caused by rheumatoid factor [34].

## 5. Conclusions

Rheumatoid factor is a kind of disease which is very harmful to human health and has high morbidity and mortality. There are many types of pathological factors in the area of rheumatic factor lesions, among which inflammatory lesions and clot formation are considered the most important. Angiogenesis is not only the material structure basis of pannus formation, but also can enrich a variety of inflammatory cells, promote inflammatory lesions, and then lead to immune blood cell damage and development. As the most important angiogenesis stimulating factor, vascular endothelial growth factor plays an indispensable role in the occurrence and development of rheumatoid factors.

In the acute stage of rheumatoid arthritis, the subsynovial membrane is mainly exudative and infiltrative, leading to endothelial cell enlargement, interstitial edema, small vessel dilatation, and neutrophil infiltration. With the development of the disease, the synovium gradually becomes thicker, forming villous protuberances, which can adhere to articular cartilage, invade cell matrix, secrete a large number of matrix metalloproteinases, and aggravate the destruction of cartilage and bone. In patients with rheumatoid arthritis, rheumatoid factors can produce stimulation, lead to vasodilation and exudation, increase vascular permeability, aggravate inflammatory edema of local tissues, and damage immune blood cell system.

Of course, with the continuous progress of modern science and technology, we have more and more understanding of diseases caused by rheumatoid factors interfering with immune blood cells, and the coping methods are constantly updated. In this paper, we have verified the harm of rheumatoid factor to human body and basically solved the problem through related treatment. In the future, the research on the treatment of rheumatoid factor induced diseases can start from controlling the activity of inflammatory cytokines through rheumatoid factor receptor inhibitors.

## Figures and Tables

**Figure 1:** Experimental inspection items.

**Figure 2:** Distribution of men and women.

**Figure 3:** Patient distribution statistics.

**Figure 4:** Changes in immune blood cell content.

**Figure 5:** Immune blood cell rheumatoid factor content.

**Figure 6:** Changes in antibodies before and after treatment.

**Figure 7:** Immune cell damage changes.

**Table 1:** Distribution of men and women.

Age	0–20	21–35	35–45	Greater than 45
Male	4	3	15	40
Female	1	2	6	29

**Table 2:** Immune blood cell changes.

	Hemoglobin content (g/l)	Red blood cells (/l)	Platelet (/l)	Rheumatoid factor (/l)
Before therapy	70	45.33	12.59	16.35
After treatment	30	21.38	7.36	12.53

**Table 3:** Patients' antibody changes.

	Number of antibodies	Number of antigens	Male	Female
Before therapy	26	52	62	38
After treatment	55	77	55	27

**Table 4:** Immune cell damage.

	Average *P* value	Average male *P* value	Average female *P* value
Before therapy	17.64	18.33	16.72
After treatment	12.21	11.95	12.56

## Data Availability

The data that support the findings of this study are available from the corresponding author upon reasonable request.
